# Analysis of Clinical Characteristics and Influencing Factors for H-Type Hypertension Complicated with Other Chronic Diseases in a Community in Beijing

**DOI:** 10.1155/2022/6974065

**Published:** 2022-09-15

**Authors:** Tianlong Li, Chen Wang, Li Ma

**Affiliations:** ^1^School of General Practice and Continuing Education, Capital Medical University, Beijing 100069, China; ^2^Department of General Medicine, Wanping Community Health Service Center, Fengtai District Beijing, Beijing 100165, China; ^3^Department of General Medicine, Beijing Tiantan Hospital, Capital Medical University, Beijing 100070, China

## Abstract

**Objective:**

The aim of the study is to analyze the clinical characteristics of patients with H-type hypertension complicated with other chronic diseases in a community in Beijing and to explore the influencing factors related to the occurrence of the disease by means of a case-control study.

**Methods:**

A questionnaire was designed. 362 residents with H-type hypertension in a community in Beijing were randomly enrolled from January 2020 to December 2021. The general data and clinical indexes of the patients were collected and their clinical characteristics were analyzed. According to the complications of other chronic diseases, they were divided into the simple hypertension group (*n* = 65) and the other chronic disease group (*n* = 297). Univariate and multivariate analyses were used to analyze the influencing factors for H-type hypertension patients with other chronic diseases.

**Results:**

Among the 362 H-type hypertension patients, 21 cases were aged 35–45 years, 35 cases were aged 45–55 years, and 127 cases were aged 55–65 years. The number of patients aged ≥65 years was 179, and the number of patients aged ≥55 years accounted for the highest proportion with a constituent ratio of 85.00%. Only 65 patients were patients with simple hypertension. The remaining 297 patients were complicated with different kinds of chronic diseases. The types of chronic diseases include malignant tumors, diabetes, rheumatoid arthritis, coronary heart disease, asthma, chronic obstructive pulmonary disease, systemic lupus erythematosus, and stroke. The proportion of H-type hypertension complicated with coronary heart disease, diabetes, and stroke is higher. Among the 297 patients, most of them were local, resident, and nonagricultural patients with a constituent ratio of 89.90%, 95.96%, and 98.98%, respectively. The prevalence rate of the male was 59.60% higher than that of the female at 40.40%. The blood types B and AB were more common. 90.57% of patients were married and the proportion of body mass index (BMI) was 45.79%. 60.61% of patients had a history of smoking, 55.56% had a history of drinking, 35.02% had a regular physical examination, 14.81% had regular exercise, and 37.71% had a light diet. There were significant differences in marital status, smoking, alcohol consumption, regular exercise, and light diet between the simple hypertension group and the chronic disease group (*P* < 0.05). The results of the logistic regression analysis showed that smoking, drinking, little exercise, and not eating lightly were the independent risk factors for other chronic diseases (*P* < 0.05).

**Conclusion:**

The incidence of H-type hypertension is higher in people ≥55 years old. Most of them are accompanied by three other chronic diseases: smoking, drinking, little exercise, and no light diet are also risk factors for chronic diseases.

## 1. Introduction

Hypertension is one of the most common clinical cardiovascular and cerebrovascular diseases, which is the most important risk factor for premature death worldwide. At present, there are about 245 million hypertensive patients in my country, accounting for more than 80% of the total number of patients with cardiovascular diseases [1, 2]. Survey data show that the prevalence of hypertension in my country is high and the control rate is low, and the prevalence of hypertension increases with age [3]. With the accelerated aging of the population in China, the number of patients with hypertension is increasing, and the morbidity and disability rates of related diseases remain high [4]. Many studies have released that hypertension is an important risk factor for stroke, which is the first cause of death and disability in adults [5]. Therefore, strengthening the prevention and control of hypertension is the focus of prevention and control of cardiovascular and cerebrovascular diseases in China.

Hypertension can be divided into two categories: consisting of primary hypertension and secondary hypertension. Clinical observation has pointed out that patients with essential hypertension are often accompanied by elevated homocysteine (Hcy), which is medically called H-type hypertension [6]. The 2010 edition of Chinese Guidelines for the Prevention and Treatment of Hypertension defines plasma Hcy ≥ 10 *μ*mol/L as an important risk factor for cardiovascular diseases. With the advancement of recent research, hyperhomocysteinaemia (HHcy) is defined as Hcy ≥ 15 *μ*mol/L in the 2018 edition of Chinese Guidelines for the Prevention and Treatment of Hypertension [7]. The increase of plasma Hcy will increase the risk of cardiovascular disease and compared with the synergistic effect of other risk factors, the risk of cardiovascular disease caused by the synergistic effect of HHcy and hypertension will further increase [8]. Previous studies have found that high Hcy can cause damage to human vascular endothelial cells, thus affecting their vascular function [9] and seriously affecting their normal physiological functions. Many studies have shown that HHcy is one of the independent risk factors for cardiovascular diseases [9, 10]. It is clearly pointed out that there is a close relationship between HHcy and the occurrence and prognosis of stroke. The prevalence rate of HHcy increases with age, and the prevalence rate of HHcy in China has increased significantly recently [11].

Compared with western countries, patients with hypertension in China often have higher Hcy levels [12]. Some scholars found that 75% of the patients with hypertension in China were H-type hypertension [13], while the data [14] from the China Stroke Primary Prevention Study(CSPPT) showed that the proportion of H-type hypertension was even higher, accounting for 80.3%. A new survey in the Suqian area showed that the prevalence rate of H-type hypertension in 873 patients with hypertension was close to 78%. There is a gender difference and the proportion of the male is significantly higher than that of the female. Gao et al. conducted a survey on H-type hypertension in the Yangquan area and showed that more than 90% of 1600 hypertensive patients were H-type hypertension, and the prevalence of the male was higher than that of the female [15]. A cross-sectional survey study found that HHcy was defined as plasma Hcy ≥16 *μ*mol/L and the incidence of HHcy in urban and rural residents in northern my country was significantly higher than that in southern China, which indicated that my country's HHcy incidence was high and there were regional differences [16]. Therefore, it is of great significance to control the progress of blood pressure and actively preventing and treating H-type hypertension to reduce the occurrence of cardiovascular events.

It can be seen that it is very necessary to study the clinical characteristics and influencing factors for H-type hypertension patients with other chronic diseases. We can find out the risk factors for H-type hypertension patients complicated with other chronic diseases and carry out targeted prevention. Thus, it is helpful to improve the prognosis of patients and protect their physical and mental health. To control the progress of blood pressure and actively preventing and treating H-type hypertension is the key to reduce the incidence of cardio-cerebrovascular events. Active analysis and research on the clinical features and factors influencing the complication of H hypertension with other chronic diseases can assist clinically to make a better prevention and treatment plan. This study investigated the patients with H-type hypertension complicated with other chronic diseases in a community in Beijing and analyzed the related factors.

## 2. Materials and Methods

### 2.1. General Information

A questionnaire was designed and 362 residents with H-type hypertension in a community in Beijing were randomly enrolled from January 2020 to December 2021. The general data and clinical indexes of the patients were collected and analyzed. The general data of patients are shown in Figures 1 and 2 and Table 1.

The diagnostic criteria of H-type hypertension were that all the selected patients met the diagnostic criteria of grade 1–3 of essential hypertension. The patients were accompanied by elevated Hcy levels ≥10 *μ*mol/L [17].

The inclusion criteria were as follows: (1) patients with type H hypertension; (2) patients over the age of 18 years; (3) patients with clear consciousness and certain reading comprehension ability; and (4) patients who were informed and gave consent to testing.

The exclusion criteria were as follows: (1) patients with secondary hypertension; (2) patients with plasma Hcy <10 *μ*mol/L; (3) patients with severe heart, brain, and renal diseases and their serious complications; (4) those with severe mental disorders; (5) those who were unable to cooperate due to various factors; (5) previous clear diagnosis of H-type hypertension and regular use of folic acid; and (6) recent use of antiepileptic drugs such as carbamazepine and phenytoin sodium.

### 2.2. Methods

#### 2.2.1. General Data Collection

The survey was carried out by the staff of a community health service center in Beijing. Moreover, the survey tool was a questionnaire on risk factors for H-type hypertension patients with other chronic diseases developed by our hospital. The questionnaire included basic personal information, lifestyle, habits, local status, permanent residence type, household type, blood type, marital status, height, weight, smoking history, waist circumference, and hip circumference. Once the questionnaires were completed, the researcher performed an audit and quality control. The questionnaire information was then entered into the hospital system by the appropriate personnel.

#### 2.2.2. Collection of Clinical Indicators

After the patient signed the informed consent form, their blood samples were taken for testing on the same day after the start of the trial. The test indicators included systolic blood pressure, diastolic blood pressure, height, weight, BMI, waist circumference, hip circumference, and blood biochemical indicators. Carotid artery thickness was measured by carotid ultrasonography on the same day after the start of the trial.

### 2.3. Statistical Analysis

The data of this test were processed and analyzed by an IBM SPSS Statistics for Windows, version 26 (IBM Corp., Armonk, NY., USA) software. The general data of patients were analyzed by a descriptive analysis and a univariate analysis was carried out by the Chi 2 test. The clinical indexes were expressed by mean ± standard deviation ($\bar{x}$ ± s). The independent sample *T* test was used for comparison between the two groups. A multivariate analysis was performed by binary logistic regression analysis with *α* = 0.05 as the test level. *P* < 0.05 was statistically significant.

## 3. Results

### 3.1. The General Data of Patients with H-Type Hypertension

#### 3.1.1. Age Statistics

First, the age statistics of the patients were analyzed. Among the 362 H-type hypertension patients, 21 cases were aged 35–45 years old and 35 cases were aged 45–55 years old. The number of patients aged 55 to 65 years was 127 and the number of patients aged ≥65 years was 179. The patients more than 55 years old accounted for the highest proportion with a composition ratio of 85.00%.

#### 3.1.2. The Clinical Characteristics of HD Hypertensive Patients with a History of Other Chronic Diseases

362 patients with H-type hypertension had a history of other chronic diseases. Only 65 patients had simple hypertension and the remaining 297 patients were complicated with different types of chronic diseases. Among them, 95 patients were complicated with 1 chronic disease, 161 patients with two kinds of chronic disorders, and 41 patients with three chronic disorders. In this study, there were 65 cases of simple H-type hypertension. H-type hypertension complicated with other types of chronic diseases were as follows: coronary heart disease (*n* = 238), diabetes (*n* = 190), stroke (*n* = 55), COPD32 (*n* = 18), asthma (*n* = 18), benign prostatic hyperplasia (*n* = 11), systemic lupus erythematosus (*n* = 7), rheumatoid arthritis (*n* = 9), thyroid carcinoma (*n* = 10), lung cancer (*n* = 3), and breast cancer (*n* = 3). From the aforementioned data, the proportion of H-type hypertension complicated with coronary heart disease, diabetes, and stroke is higher.

Among the 297 patients with H-type hypertension, most of them were local, resident, and nonagricultural patients with a constituent ratio of 89.90%, 95.96%, and 98.98%, respectively. The prevalence rate of the male was 59.60%, which was higher than that of the female at 40.40%. The blood types B and AB were more common and 90.57% of the patients were married. Based on the BMI classification, most of the patients were normal, accounting for 45.79%. 60.61% of the patients had a history of smoking, 55.56% had a history of drinking, 35.02% had regular physical examinations, 14.81% had regular exercise, and 37.71 had a light diet.

### 3.2. Mono-Factor Analysis of Chronic Diseases in Patients with H-Type Hypertension

A univariate analysis is performed on the related factors for chronic diseases in patients with H-type hypertension as shown in in Table 2. The results showed the gender, resident type, local, household, blood type, BMI grade, smoking history, and alcohol consumption of the two groups of patients. There were no significant differences in general data such as history, regular physical examination, regular exercise, and light diet (*P* > 0.05). There were significant differences in the marital status and whether to use enalapril maleate folic acid tablets between the simple hypertension group and the combined chronic disease group (*P* < 0.05).

### 3.3. Clinical Detection Indexes between the Simple Hypertension Group and Patients with Chronic Disease Group

The clinical indicators of patients with simple hypertension and those with chronic diseases are compared in Table 3. The results showed that clinical indicators had no statistical difference (*P* > 0.05).

### 3.4. Multivariate Analysis of Variance Affecting Chronic Diseases in Patients with H-Type Hypertension

Logistic regression analysis was performed on the factors affecting H-type hypertension patients with chronic diseases. The relevant indicators with a statistical significance (*P* < 0.05) in the univariate analyses were substituted into the logistic regression model for analysis. Whether the patients had other chronic diseases was the factor. The results showed that smoking, drinking, little exercise, and no light eating were the independent risk factors for the combination of other chronic diseases (*P* < 0.05). All results are shown in Table 1.

## 4. Discussion

HHcy is a type of disease characterized by increased levels of Hcy6 in the blood. Many studies have found that HHcy can damage vascular endothelial cells and cause changes in the vascular structure. It leads to vascular dysfunction, resulting in hypertension and vascular disease, which is an independent risk factor for atherosclerosis and is closely related to the occurrence of cardiovascular and cerebrovascular diseases. Epidemiological studies have also proved [18] that the incidence of cardiovascular events in hypertensive patients with HHcy is about 5 times higher than that in pure hypertensive patients [18]. Men with H-type hypertension had an approximately 12-fold increased risk of cardiovascular events and women with H-type hypertension had an approximately 28-fold increased risk of cardiovascular events. It can be seen that it is still of great significance to formulate effective and effective prevention and treatment plans as soon as possible to improve the prognosis of such patients.

The results are consistent with previous research reports [19]. The reason may be that the risk of male exposure to adverse risk factors is higher than that of females. In addition, the blood types B and AB were more common, of which 90.57% were married, and most of them were normal in BMI classification, accounting for 60.61% of patients had a history of smoking, 55.56% had a history of drinking, 35.02% had a regular physical examination, 14.81% had regular exercise, and 37.71% had a light diet, respectively.

Many studies have shown that the levels of blood pressure, blood sugar, blood lipids, and D-dimer are closely related to the occurrence of cardiovascular and cerebrovascular events [20]. Early study has suggested the incidence of stroke in both the intervention group and the control cohort increases with the increase in blood pressure, and the risk of stroke is positively correlated with the level of increased blood pressure [21]. Yu Jinming et al. pointed out that the blood pressure fluctuation of stroke-hypertensive patients during the follow-up period was significantly higher than that of stroke-free hypertensive patients and the risk of stroke increased with the increase of blood pressure fluctuation. Under the same conditions, the risk of stroke is also high when the average blood pressure and baseline blood pressure fluctuate widely [22].

In this study, univariate and multivariate analysis methods were used for analysis. This is inconsistent with the conclusions of previous research reports. The reason might be that the patients included were older and most of them were residents. The sample type was relatively single and the sample size in the simple hypertension group was relatively small with a certain bias.

In this study, there were 65 cases of simple H-type hypertension. The proportion of H-type hypertension complicated with coronary heart disease, diabetes, and stroke is higher. This suggests that H-type hypertension may be associated with the abovementioned diseases, but this needs to be confirmed by further research studies. In this study, there were significant differences in marital status, smoking, alcohol consumption, regular exercise, and light diet between the simple hypertension group and the chronic disease group (*P* < 0.05). Generally speaking, in the comparison between the two groups, the probability of chronic disease in married patients was higher than that of unmarried and divorced, while in the comparison between the groups, the proportion of married patients with chronic diseases was higher than that of those without chronic diseases. One of the reasons why married patients with hypertension are more likely to develop chronic diseases is that they are older and have poorer physical quality. The other may be due to the influence of mental factors. Married people tend to have more mental stress and do not pay enough attention to their own illness. The mental state will affect the physical state. Bad living habits also have a great negative impact on the control of patients' diseases; therefore, medical staff should pay attention to understand their living conditions when intervening with patients and helping them correct their wrong habits and develop a healthy lifestyle.

To sum up, most of the patients with H-type hypertension in a community in Beijing are complicated with three other chronic diseases. Scientific and reasonable prevention and therapeutic strategies need to be made to improve the prognosis of the patients. The type of sample included in this study is relatively single, and the sample size is relatively small, which still needs to be further expanded to confirm the accuracy of the conclusion.

## 5. Conclusion

The incidence of H-type hypertension is higher in people ≥55 years old. Most of them are accompanied by three other chronic diseases. Smoking, drinking, little exercise, and no light diet are also risk factors for chronic diseases. General practitioners need to pay more attention to these risk factors.

## Figures and Tables

**Figure 1:** Age statistics of patients with H-type hypertension.

**Figure 2:** Statistics on the history of other chronic diseases at the same time.

**Table 1:** Logistic regression analysis of chronic diseases in patients with H-type hypertension.

Factors	*β* value	SE	Wald value	*P* value	OR value (95 CI)
Marital status	0.371	0.314	1.396	0.237	1.449 (0.783∼2.682)
Smoking	0.822	0.291	7.979	0.005	2.275 (1.286∼4.024)
Drink alcohol	0.840	0.301	7.788	0.005	2.316 (1.284∼4.179)
Regular exercise	0.799	0.289	7.644	0.006	2.223 (1.262∼3.917)
Light diet	0.847	0.311	7.417	0.006	2.333 (1.268∼4.291)

**Table 2:** Mono-factor analysis of chronic diseases in patients with H-type hypertension (*n*/%).

Project	Total number (*n* = 362)	Simple hypertension group (*n* = 65)	Group with chronic diseases (*n* = 297)	*χ* ^2^	*P*
*Gender*				1.449	>0.05
Female	151	31 (47.69)	120 (40.40)		
Male	211	34 (52.31)	177 (59.60)		

*Local/nonlocal*				1.937	>0.05
Local	329	62 (95.38)	267 (89.90)		
nonlocal	33	3 (4.62)	30 (10.10)		

*Resident type*				0.306	>0.05
Household registration	348	63 (96.92)	285 (95.96)		
Nonhousehold registration	9	1 (1.54)	8 (2.69)		
Unknown	5	1 (1.54)	4 (1.35)		

*Household separation*				2.121	>0.05
Agriculture	8	3 (4.62)	5 (1.68)		
Nonagricultural	354	62 (95.38)	292 (98.98)		

*Blood type*				2.339	>0.05
A type	76	6 (9.23)	35 (11.78)		
B type	115	20 (30.77)	95 (31.99)		
AB type	120	19 (29.23)	101 (34.01)		
O type	51	20 (30.77)	66 (22.22)		

*Marital status*				31.910	<0.05
Unmarried	13	10 (15.38)	3 (1.01)		
Married	320	51 (15.94)	269 (90.57)		
Divorce	29	4 (6.15)	25 (8.42)		

*BMI grading*				3.454	>0.05
Too light	3	1 (1.54)	2 (0.67)		
Overweight	108	25 (38.46)	83 (27.95)		
Normal	161	25 (38.46)	136 (45.79)		
Obesity	90	14 (21.54)	76 (25.59)		

*Smoking*				10.648	<0.05
Yes	205	25 (38.46)	180 (60.61)		
No	157	40 (61.54)	117 (39.39)		

*Alcohol consumption*				4.207	<0.05
Yes	192	27 (41.54)	165 (55.56)		
No	170	38 (58.46)	132 (44.44)		

*Regular physical examination (>1/year)*				0.032	>0.05
Yes	126	22 (33.85)	104 (35.02)		
No	236	43 (66.15)	193 (64.98)		

*Regular exercise (>5 times/week, >30 min/times)*				9.327	<0.05
Yes	64	20 (30.77)	44 (14.81)		
No	298	45 (69.23)	253 (85.19)		

*Light diet*				9.463	<0.05
Yes	150	38 (58.46)	112 (37.71)		
No	212	27 (41.54)	185 (62.29)		

**Table 3:** Clinical detection indexes between the simple hypertension group and the chronic disease group ($\bar{x}$ ± s).

Project	Simple hypertension group (*n* = 65)	Group with chronic diseases (*n* = 297)	*T*	*P*
Systolic blood pressure (mmHg)	127.63 ± 31.87	126.65 ± 32.38	0.222	>0.05
Diastolic pressure (mmHg)	76.93 ± 23.07	76.72 ± 23.38	0.066	>0.05
Height (cm)	162.87 ± 12.13	158.29 ± 19.71	1.799	>0.05
Body weight (kg)	65.81 ± 16.19	66.22 ± 17.21	0.176	>0.05
BMI (kg/m^2^)	24.71 ± 4.30	26.43 ± 8.25	1.632	>0.05
Waist circumference (cm)	85.03 ± 7.37	88.84 ± 15.29	1.958	>0.05
Hip circumference (cm)	92.93 ± 7.07	98.41 ± 33.83	1.298	>0.05
Na (mmol/L)	141.57 ± 2.43	141.61 ± 5.09	0.062	>0.05
Cl (mmol/L)	105.15 ± 3.35	104.63 ± 9.57	0.432	>0.05
Ca (mmol/L)	2.21 ± 0.08	2.19 ± 0.27	0.591	>0.05
P (mmol/L)	1.15 ± 0.35	1.21 ± 0.39	1.143	>0.05
CO_2_ (mmol/L)	24.49 ± 2.41	24.36 ± 3.74	0.268	>0.05
SdLDL-C (mmol/L)	1.03 ± 1.32	1.09 ± 1.53	0.293	>0.05
TP (g/L)	72.74 ± 9.56	73.88 ± 11.42	0.749	>0.05
ALB (g/L)	44.31 ± 1.98	43.87 ± 6.78	0.518	>0.05
BUN (mmol/L)	5.28 ± 2.02	5.41 ± 4.53	0.226	>0.05
CREA (*μ*mol/L)	85.06 ± 49.94	77.01 ± 40.65	1.385	>0.05
UA (mmol/L)	345.26 ± 310.06	327.52 ± 337.43	0.389	>0.05
TG (mmol/L)	1.71 ± 0.68	1.83 ± 0.89	1.023	>0.05
CHO (mmol/L)	4.44 ± 2.47	4.87 ± 3.19	1.021	>0.05
HDL-C (mmol/L)	1.51 ± 0.75	1.54 ± 0.85	0.263	>0.05
LDL-C (mmol/L)	2.65 ± 1.83	2.69 ± 2.22	0.135	>0.05
TBIL (*μ*mol/L)	14.32 ± 4.18	15.45 ± 10.83	0.827	>0.05
ALT (U/L)	24.86 ± 18.66	22.71 ± 15.21	0.989	>0.05
AST (U/L)	25.16 ± 5.84	26.02 ± 8.73	0.758	>0.05
LDH (U/L)	152.62 ± 42.68	165.99 ± 88.01	1.193	>0.05
HBDH (U/L)	136.02 ± 44.08	140.84 ± 53.14	0.682	>0.05
CK (U/L)	96.39 ± 75.21	91.55 ± 73.15	0.481	>0.05
CKMB (U/L)	17.93 ± 8.07	17.86 ± 13.23	0.041	>0.05
ALP (U/L)	67.74 ± 24.56	70.27 ± 28.49	0.664	>0.05
GGT (U/L)	34.49 ± 11.81	33.45 ± 17.82	0.449	>0.05
K (mmol/L)	4.49 ± 0.91	4.47 ± 1.13	0.133	>0.05
GFR (mL/min/1.73 m^2^)	72.72 ± 21.86	72.62 ± 28.31	0.027	>0.05
Carotid intima thickness (mm)	1.89 ± 1.21	2.28 ± 2.22	1.371	>0.05

CO_2_: carbon dioxide; Sd LDL-C: small dense low-density lipoprotein cholesterol; TP: protein total; ALB: albumin; BUN: blood urea Nitrogen; CREA: creatinine; UA: uric acid; TG: triglycerides; CHO: cholesterol determination; HDL-C: high-density lipoprotein cholesterol; LDL-C: low-density lipoprotein cholesterol; TBIL: bilirubin total; ALT: alanine transaminase; AST: aspartate transaminase; LDH: lactate dehydrogenase; HBDH: hydroxybutyrate dehydrogenase; CK: creatine kinase; CKMB: creatine kinase isoenzyme; ALP: alkaline phosphatase; GGT: gamma-glutamine acylase; GFR: glomerular filtration rate.

## Data Availability

The data that support the findings of this study are available on request from the corresponding author upon reasonable request.
